The article "Lung Cancer Radiotherapy: Simulation and Analysis Based on a Multicomponent Mathematical Model" was published in 2021. Journal: Comput Math Methods Med.

# Lung Cancer Radiotherapy: Simulation and Analysis Based on a Multicomponent Mathematical Model

**DOI:** 10.1155/2021/6640051

**Published:** 2021-04-29

**Authors:** Wen-song Hong, Shun-guan Wang, Gang-qing Zhang

**Affiliations:** Radiotherapy Department of Guangdong Second Provincial General Hospital, Guangzhou 510317, China

## Abstract

**Background:**

Lung cancer has been one of the most deadly illnesses all over the world, and radiotherapy can be an effective approach for treating lung cancer. Now, mathematical model has been extended to many biomedical fields to give a hand for analysis, evaluation, prediction, and optimization.

**Methods:**

In this paper, we propose a multicomponent mathematical model for simulating the lung cancer growth as well as radiotherapy treatment for lung cancer. The model is digitalized and coded for computer simulation, and the model parameters are fitted with many research and clinical data to provide accordant results along with the growth of lung cancer cells in vitro.

**Results:**

Some typical radiotherapy plans such as stereotactic body radiotherapy, conventional fractional radiotherapy, and accelerated hypofractionated radiotherapy are simulated, analyzed, and discussed. The results show that our mathematical model can perform the basic work for analysis and evaluation of the radiotherapy plan.

**Conclusion:**

It will be expected that in the near future, mathematical model will be a valuable tool for optimization in personalized medical treatment.

## 1. Background

Lung cancer may be one of the most deadly killers in our world. According to the global cancer statistics 2018, it was estimated that there were about 2 million new lung cancer cases as well as 1.7 million death cases in 2018 all over the world, both incidence and mortality stood in the first place [1]. In the subtype, non-small cell lung cancer (NSCLC) was in the absolute dominance (85%). Although there were many new technologies for diagnosis and treatment of lung cancer, the five-year survival was still in a very low level (10-20%) [2].

Radiotherapy (RT) is a valuable approach for lung cancer treatment, especially for local advanced lung cancer [3, 4]. A serial of clinical evidences elucidate that radiotherapy combined with chemotherapy or immunotherapy may improve the local control of lung cancer [5–7]. In recent years, a special radiotherapy method, named stereotactic body radiotherapy (SBRT), has been introduced to alternative treatment for early stage inoperable NSCLC [8–10]. In SBRT, a lot of small radiation beams are delivered exactly to the tumor target in one or several fractions. Many international cooperative group trails have confirmed that SBRT can return high rates of tumor control without severe toxicity [11, 12].

Mathematical model has been utilized to expound the physiological and pathological processing of human being for a long time. For example, as early as 1960s, Priore made an attempt to evaluate the human tumor response to chemotherapy with a mathematical model [13]. In this decade, mathematical models were extended to many fields of medical research dramatically. In 2015, Michor and Beal provided detailed analysis on mathematical modeling for cancer treatment improvement [14]. In addition, a serial of papers about mathematical modeling for precision medicine, impact of vaccine, and prediction of cancer drug resistance were presented by many researchers [15–17]. Because of the complicacy of physiology and pathology, there were a lot of different mathematical representations for emulating the realistic processing, such as logistic model, ordinary differential equation (ODE) model, and stochastic differential equation (SDE). As the superiority of simplicity and stability, the ODE model has been widely used in the fields of infection control, pharmacodynamics, and tumor metabolism [18–21]. In our past work, we have developed a mathematical model based on ODE for tumor radiotherapy [22]. So, the model in this paper is elicited in ODE format.

In this paper, we constitute an ODE model for emulating the processing of tumor growth and tumor radiotherapy. It is supposed in our model that the tumor colony, even in the same colony, may have very different features such as growth speed, apoptosis time, and drug resistance and radiation sensitivity, so a hypothesis of multicomponent structure should be eligible [23]. In order to lead some further applications to clinical research, we feed our model parameters with the data refined from many clinical studies of lung cancer; furthermore, numerical simulation and analysis were performed based on our own developed computer codes.

The paper is organized as follows: firstly, the tumor growth model and tumor radiotherapy model are listed in detail. Then, the outputs of numerical simulation were figured out with corresponding analysis and explanation. Finally, a discussion is worked out.

## 2. Methods

### 2.1. Tumor Growth Model

Many mathematical models of tumor growth have been applied in basic or clinical research [24], among which the logistic model (LM) and Gompertz model (GM) may be the most popular. LM is formulated as

(1) $$\begin{array}{c} \frac{dV}{dt}=aV\left(1-\frac{V}{K}\right), \end{array}$$

where *V*, a function of time *t*, is the tumor volume and *d*/*dt* is the derivative formula with respect to *t*. Both *a* and *K* are constant related to tumor proliferation kinetics and carrying capacity, respectively.

GM was proposed first by Benjamin Gompertz in 1925 [25]. The model is described as

(2) $$\begin{array}{c} \frac{dV}{dt}=aV-bV\ln V, \end{array}$$

where *a* and *b* are coefficients.

It can be deduced that because of the carrying capacity *K* in (1), the leap for Gompertz model will be larger.

As we know, the tumor growth is impacted by many natural factors, such as nutrient, the tumor cell cycle, and even the contest between the neighbor tumor cells. Also in the same tumor colony, the cells may be at different states and have different growth rates, for example, active tumor and quiescent cells. So we can conclude the following model rationally (Figure 1 and formula (3)):

(3) $$\begin{array}{c} \left\{\begin{array}{c} \frac{dV_{1}}{dt}=a_{1}V_{1}\left(1-\frac{V_{1}}{K_{1}}\right)+p_{Q1}V_{Q}-\left(p_{1Q}+p_{1ND}\right)V_{1}\\ \frac{dV_{2}}{dt}=a_{2}V_{2}\left(1-\frac{V_{2}}{K_{2}}\right)+p_{Q2}V_{Q}-\left(p_{2Q}+p_{2ND}\right)V_{2}\\ \vdots \\ \frac{dV_{m}}{dt}=a_{m}V_{m}\left(1-\frac{V_{m}}{K_{m}}\right)+p_{Qm}V_{Q}-\left(p_{mQ}+p_{mND}\right)V_{m}\\ \frac{dV_{Q}}{dt}=\left(p_{1Q}V_{1}+p_{2Q}V_{2}+\cdots +p_{mQ}V_{m}\right)-\left(p_{Q1}+p_{Q2}+\cdots +p_{Qm}+p_{QND}\right)V_{Q}\\ \frac{dV_{ND}}{dt}=p_{1ND}V_{1}+p_{2ND}V_{2}+\cdots +p_{mND}V_{m}+p_{QND}V_{Q}-\eta V_{ND}\\ m=1,2,\cdots ,M, \end{array}\right. \end{array}$$

where *V*_*m*_ is the volume of the active tumor *T*_*m*_ mentioned in Figure 1. *η* is the clear rate of nondividing cells into blood. Here, we prefer the LM tumor growth model.

### 2.2. Tumor Radiotherapy Model

The most popular model for tumor radiotherapy may be the linear-quadratic (LQ) model [26]. In the LQ model, it is assumed that the X-ray can break the double-stranded DNA of the tumor cells and lead to the death of them. The probability of the tumor cell death is related to the dose of the given X-rays, while the survival probability of the tumor cells can be described as

(4) $$\begin{array}{c} S=e^{-\alpha D-\beta D^{2}}, \end{array}$$

where *S* is the probability of survival tumor cells, *D* is single radiation dose, *e* is the natural constant, and *α*, *β* are the parameters relating to the radiation sensitivity, which is represented as *α*/*β*. For using in this paper, we rewrite formula (4) in an ODE formulation:

(5) $$\begin{array}{c} \frac{dV}{dt}=-\left(\alpha D+2\beta D^{2}\right)V. \end{array}$$

Here, *D* is the radiation dose rate. Because X-ray acts as breaking the double-stranded DNA and stopping proliferation of the cells, it can impact the active and quiescent cells only, but not the nondividing cells. Then, the single-dose radiotherapy model can be

(6) $$\begin{array}{c} \left\{\begin{array}{c} \frac{dV_{1}}{dt}=a_{1}V_{1}\left(1-\frac{V_{1}}{K_{1}}\right)+p_{Q1}V_{Q}-\left(p_{1Q}+p_{1ND}\right)V_{1}-\left(\alpha_{1}D+2\beta_{1}D^{2}\right)V_{1}\\ \frac{dV_{2}}{dt}=a_{2}V_{2}\left(1-\frac{V_{2}}{K_{2}}\right)+p_{Q2}V_{Q}-\left(p_{2Q}+p_{2ND}\right)V_{2}-\left(\alpha_{2}D+2\beta_{2}D^{2}\right)V_{2}\\ \vdots \\ \frac{dV_{m}}{dt}=a_{m}V_{m}\left(1-\frac{V_{m}}{K_{m}}\right)+p_{Qm}V_{Q}-\left(p_{mQ}+p_{mND}\right)V_{m}-\left(\alpha_{m}D+2\beta_{m}D^{2}\right)V_{m}\\ \frac{dV_{Q}}{dt}=\left(p_{1Q}V_{1}+p_{2Q}V_{2}+\cdots +p_{mQ}V_{m}\right)-\left(p_{Q1}+p_{Q2}+\cdots +p_{Qm}+p_{QND}\right)V_{Q}-\left(\alpha_{Q}D+2\beta_{Q}D^{2}\right)V_{Q}\\ \frac{dV_{ND}}{dt}=p_{1ND}V_{1}+p_{2ND}V_{2}+\cdots +p_{mND}V_{m}+p_{QND}V_{Q}-\eta V_{ND}\\ m=1,2,\cdots ,M. \end{array}\right. \end{array}$$

Now in the routine radiotherapy practice, the radiation dose may be divided into many fractions, for example, a larger dose fractional radiotherapy may have several fractions, while normal fractional radiotherapy may take 30 times in one treatment course, and each fraction may take only several or dozens of minutes for radiation. To simulate this process, a piecewise integration equation is presented here:

(7) $$\begin{array}{c} V_{1}=\overset{L}{\underset{i=1}{\sum }}\left(\begin{array}{c} \int_{t_{0}}^{t_{F}}\left(a_{1}V_{1i}\left(1-\frac{V_{1i}}{K_{1}}\right)+p_{Q1}V_{Qi}-\left(p_{1Q}+p_{1ND}\right)V_{1i}\right)dt\\ -\left(\int_{t_{0}}^{t_{R}}\left(\left(\alpha_{1}D_{i}+2\beta_{1}{D_{i}}^{2}\right)V_{1i}\right)dt\right) \end{array}\right), \end{array}$$

where *L* is the total fraction number in one radiotherapy course, (*t*_0_,  *t*_*F*_) is the time interval between each two fractions, (*t*_0_,  *t*_*R*_) is the radiation time, and the subscript *i* in *V*_1*i*_, *V*_*Qi*_, *D*_*i*_ indicates that *V*_1_, *V*_*Q*_, and *D* are in the *i*^th^ fraction, respectively. According to formula (6), the equations of *V*_1_, *V*_2_, *V*_*m*_, and *V*_*Q*_ can be built in the same way like that of *V*_1_.

### 2.3. Parameters of the Model

To simplify the simulation process, we set the parameter *M* in (6) to 2; then, the active tumor cell colony is comprised of 2 kinds, *T*_1_ and *T*_2_ with the volume *V*_1_ and *V*_2_, respectively, and also, it is assumed that the dose rate *D*_*i*_ in each fraction be a constant *D*.

Much research has been done for fitting the tumor model parameters with clinical data [27, 28]. In 2013, Benzekry et al. recorded a serial of comprehensive experiments for several classical mathematical models for tumor growth [29]; in their paper, the parameters in many mathematical models include LM and GM for lung and breast cancer are been fitted with the experimental data. As a key reference, their lung data was extracted for estimating and fitting the parameters of our tumor growth model; also, we refined our model parameters according to the dada of the volume double time of lung cancer in some studies [30, 31].

The parameters in LQ mode are mainly about the value of *α* and *β*. It was recommended in many paper that the value of *α*/*β* for lung cancer can be taken from 10 to 20 for clinical use [32, 33]; moreover, in paper [34], the value of *α*/*β*, estimated from 1294 data of non-small cell lung cancer patients treated with stereotactic body radiotherapy, could be in the range of 12-16. We referred their papers for fitting the parameters of LQ model registered in this paper.

In order to give the quantitative assessment of the radiotherapy effectiveness, a treatment ratio is introduced as

(8) $$\begin{array}{c} \text{Treatment ratio}=\text{Tumor volume after RT}/\text{Tumor volume before RT}. \end{array}$$

This is the metric for evaluating the treatment effect of RT, the lower the better.

The crucial model parameters in this paper are listed in Table 1.

### 2.4. Programming and Processing

The computer programming codes are developed for simulating and processing. The development tools are MATLAB R2018a (MathWorks Corporation, Natick, MA, USA) and Visual Studio Professional 2012 (Microsoft Corporation, Redmond, Washington, USA).

## 3. Numerical Simulation and Analysis

### 3.1. Analysis of Tumor Growth Model

The simulation results of GM, LM, and our MCM are all plotted in Figure 2. As references, any experimental data extracted from the studies of the growth of A549 cell lines, which belong to human NSCLC [35], are also presented here. The results reveal that all the models present a good coincidence at the beginning of the tumor growth. In some research, the experiments of tumor growth had given the evidence that GM and LM could return the perfect curves along with the experimental data during the first 20 days, but in the following days, their fitting power would be more and more poor [29]. Because of the simple representations and unchangeable coefficients, it might be the essential inextricability for these models to hold the real data entirely, while in our MCM, some parameters can be adjusted easily for adapting the curves as much as possible to the real data (A549 in Figure 2(a)).

### 3.2. Analysis of SBRT

In 2018, an evidence-based guideline was produced by the American Society for Radiation Oncology (ASTRO) on treatment for early stage NSCLC patient with SBRT [36]. In additional, many clinical trials were performed to compare the treatment results between SBRT and surgery. For example, the data of posttreatment mortality after SBRT and surgery drawn out by William et al. gave a supportive evidence that SBRT might have lower mortality than surgery [18].

There are many fractional dose approaches for SBRT treatment. The fraction may be 1 to 10, and the dose per fraction may be 7 Gy to 23.5 Gy, according to the tumor size, tumor place, and so on. Some typical values from the references are picked out to analyze the results through our MCM (Figure 3).

From the simulating results, we can find that all the four plans have the perfect feedback on tumor control. Among them, 48 Gy/4 Fr and 60 Gy/8 Fr may be better, but the dose per fraction of 12 Gy or total dose of 60 Gy will cause more toxicity to the normal tissues. The other two plans have similar scores of tumor control enough for clinical practice, so it may be the most reasonable plan for 50 Gy/5 Fr to SBRT.

### 3.3. Analysis of Conventional Fractional RT (CFRT)

CFRT has a long history for lung cancer treatment, especially for advanced one. From anterior-posterior two fields RT, multifields conformal RT to intensity-modulated RT (IMRT), CFRT plays a crucial role in the improvement of lung cancer therapy. Although there are not any evidences that CFRT can improve the survival rate of lung cancer significantly, it has the effectiveness in local control and symptom relief; moreover, it can give the patients an alternative approach to help them to struggle against the cancer. In 2013, Aileen et al. found in their surveys that many patients with incurable lung cancer released more positive expectations about RT [37].

In the clinical practice, CFRT may have about 30~35 fractions and 1.8~2.2 Gy per fraction, 5 fractions per week. ASTRO also recommended in the guideline in 2015 that for treatment of locally advanced NSCLC with curative-intent, the RT dose-fractionation should be 60 Gy given in 2 Gy per fraction [3]. But in the simulating result (Figure 4), we can find that although the plan of 60 Gy/30 Fr can do well to higher *α*/*β* tumor *T*_2_ (Figure 4(a)), its control power to low *α*/*β* tumor *T*_1_ may be incompetent, even the total dose rises to 70 Gy (Figure 4(b)), while if we raise the dose per fraction to 2.5 Gy (Figure 4(c)), the result may improve significantly. It should be an encouraging hint for us to get better tumor control by changing only the dose per fraction while keeping the same total dose of RT; this may be the theoretical support to hypofractionated RT (HFRT).

### 3.4. Analysis of Accelerated Hypofractionated RT

Along with the development of RT technique, there are many improvements on CFRT for lung cancer, such as HFRT. It was reported that the proliferation of tumor cells of NSCLC could accelerate in 3-4 weeks after the beginning of RT [38]; in order to minimize the impact of the proliferation, the dose per fraction was recommended to rise to 2.5 to 3.0 Gy; then, the total treatment time decreased correspondently. Here, HFRT was elicited. But larger single dose could cause more harm to normal tissue, so it was rational to reduce the dose per fraction as well as increase the fractions per day. Usually the plan was 1.2~1.5 Gy per fraction while 2 fractions per day, 5 days a week, but the plan was not mandatory; there was also an HFRT plan containing 1.5 Gy per fraction at 3 fractions a day [39]. A good amount of research reported that HFRT could achieve local control improvement without increasing toxicity [40–42]; however, there was still no comprehensive comparative outcome of the different HFRT plans.

As showing in Figure 5(a) and comparing with Figure 4(b), when we only change the RT fractions from 1 per day to 2 per day, we will receive a perfect response that the treatment ratio about *T*_1_ drops dramatically from 0.240 to 0.0065. It can be concluded from Figure 5 that if we can find out the proliferation of the surrounding normal tissues of the tumor, we can reach an optimization of HFRT just for adjusting the fraction gap of HFRT.

## 4. Discussion

Everything may have its own rules, without exception. The most important thing should be how accurate and simple we can describe the rules. Mathematical model has been proven to be a succinct and powerful tool in the fields of nature phenomena analysis. For tumor metabolism, with a proper mathematical model and any partial data, we can analyze the past state of the tumor as well as its future development. For example, in our MCM, once the model is reconstructed with the in vivo data, we can work out a serial of specific parameters to give the evaluation and prediction of the tumor growth; in addition, we can also build a bridge between the tumor and the blood components, because the nondividing tumor cells (*T*_*m*_) will be cleared and broken down in to the blood eventually. If some biochemicals taken from the blood test are confirmed to come from a curtain tumor, then the tumor features can be further analyzed according to the biochemicals and the tumor mathematical model. This is to say that we can do quantitative analysis about all the active tumors (*T*_1_, *T*_2_, and *T*_*m*_) through the blood test of the patients.

As we know, it will be a more complicated and time-consuming work to find a new approach for treatment of a specific illness. We have to repeat a serial of endless experiments until a result, maybe a failure result, is returned. Will there be a shortcut? Perhaps, mathematical model may be the one. For tumor radiotherapy, with the support of mathematical model, as soon as the treatment hypothesis is proposed, we can give it the first feasible evaluation about the total treatment dose, the dose per fraction, and the time gap between two fractions; also, we can receive some reasonable advices from the model to optimize the treatment. The huge experiments are no more needed, and what we have to do is to wait for the answers from the computer.

As a beneficial attempt, we use our MCM to explain the dominant approaches of lung cancer radiotherapy. To SBRT, our model returns the similar results as current clinical approaches as well as recommends a feasible plan (50 Gy/5 Fr) for clinical reference. To CFRT, our model shows that a perfect tumor control cannot be reached with normal dose per day (2 Gy) despite of high total dose, while with higher dose per day (for example, 2.5 Gy) and normal total dose, the tumor control becomes better! Consequently, it is necessary to make an improvement from CFRT to HFRT or accelerated HFRT. An accordant conclusion is also proposed by some clinical trial [43, 44].

But this may be a dream far away from the reality. Although the artificial intelligence (AI) becomes hotter and hotter in recent years, there still has a very long and roundabout way to reach the goals of the clinical application of the mathematical model. For our MCM, the main problem may be the extraction of parameters such as *T*_1_, *T*_2_, and *T*_*m*_, as well as *α* and *β*. Anyway, the future is desirable. It must be the most imperative study for us to determine which kind of the model will be enough for explaining the biophysiological process of the tumor and the interaction between the tumor and radiation ray. It is also a heavy work to gather and analyze the experimental and clinical data for the parameters optimization of the models. These may be our coming work.

## 5. Conclusions

Tumor growth is a very complicated process. Naturally, a single tumor cell model may be too rough to explain the tumor metabolism. In our MCM, two different kinds of tumor cells are considered to analyze and evaluate the radiotherapy approaches for lung cancer treatment. The result shows that MCM has made a successful step on clinical evaluation. It should be a valuable study for further research.

## Figures and Tables

**Figure 1:** Illustration of multicomponent model of tumor growth. It is assumed that there are different tumor cells in the tumor colony: the quiescent cells, which suspend dividing and can change to active tumors and nondividing cells; nondividing cells, which are dead and waiting to be cleared into the blood; and active tumors, which can divide normally and can change to quiescent cells and nondividing cells, and the active tumor also have different types, *T*_1_, *T*_2_, ⋯*T*_*m*_. *p*_*ij*_ is the probability of cell *i* changing to cell *j*. *η* is the clear rate.

**Figure 2:** Comparison of GM, LM, and MCM.

**Figure 3:** Comparison of SBRT with different RT parameters.

**Figure 4:** Comparison of CFRT with different RT parameters.

**Figure 5:** Comparison of HFRT with different RT parameters.

**Table 1:** Crucial parameters of models.

Model	Parameter	Unit
GM	*a* = 0.743, *b* = 0.0792	Day^−1^
LM	*a* = 0.502	Day^−1^
	*K* = 1297	mm^3^
MCM	*a*_1_ = 0.862, *a*_2_ = 0.501	Day^−1^
	*K*_1_ = 1397, *K*_2_ = 1174	mm^3^
	*p*_*Q*1_ = 0.1, *p*_1*Q*_ = 0.2, *p*_1ND_ = 0.2, *p*_*Q*2_ = 0.1, *p*_2*Q*_ = 0.2, *p*_2ND_ = 0.2, *p*_*Q*ND_ = 0.09, *η* = 0.4	Day^−1^
LQ	*α*_1_ = 0.194, *α*_2_ = 0.3705, *α*_*Q*_ = 0.3	Gy^−1^
	*β*_1_ = 0.063, *β*_2_ = 0.02335, *β*_*Q*_ = 0.15	Gy^−2^

## Data Availability

All data, model, and code used in this study are available from the corresponding author by request.
